# Machine Learning-Based Ensemble Model for Zika Virus T-Cell Epitope Prediction

**DOI:** 10.1155/2021/9591670

**Published:** 2021-10-01

**Authors:** Syed Nisar Hussain Bukhari, Amit Jain, Ehtishamul Haq, Moaiad Ahmad Khder, Rahul Neware, Jyoti Bhola, Moslem Lari Najafi

**Affiliations:** ^1^University Institute of Computing, Chandigarh University, Mohali, Punjab, India; ^2^Department of Biotechnology, University of Kashmir, Srinagar, J & K, India; ^3^Applied Science University, Al Eker, Bahrain; ^4^Department of Computing, Mathematics and Physics, Western Norway University of Applied Sciences, Bergen, Norway; ^5^Electronics & Communication Engineering Department, National Institute of Technology, Hamirpur, India; ^6^Pharmaceutical Science and Cosmetic Products Research Center, Kerman University of Medical Sciences, Kerman, Iran

## Abstract

Zika virus (ZIKV), the causative agent of Zika fever in humans, is an RNA virus that belongs to the genus *Flavivirus*. Currently, there is no approved vaccine for clinical use to combat the ZIKV infection and contain the epidemic. Epitope-based peptide vaccines have a large untapped potential for boosting vaccination safety, cross-reactivity, and immunogenicity. Though many attempts have been made to develop vaccines for ZIKV, none of these have proved to be successful. Epitope-based peptide vaccines can act as powerful alternatives to conventional vaccines due to their low production cost, less reactogenic, and allergenic responses. For designing an effective and viable epitope-based peptide vaccine against this deadly virus, it is essential to select the antigenic T-cell epitopes since epitope-based vaccines are considered safe. The in silico machine-learning-based approach for ZIKV T-cell epitope prediction would save a lot of physical experimental time and efforts for speedy vaccine development compared to *in vivo* approaches. We hereby have trained a machine-learning-based computational model to predict novel ZIKV T-cell epitopes by employing physicochemical properties of amino acids. The proposed ensemble model based on a voting mechanism works by blending the predictions for each class (epitope or nonepitope) from each base classifier. Predictions obtained for each class by the individual classifier are summed up, and the class with the majority vote is predicted upon. An odd number of classifiers have been used to avoid the occurrence of ties in the voting. Experimentally determined ZIKV peptide sequences data set was collected from Immune Epitope Database and Analysis Resource (IEDB) repository. The data set consists of 3,519 sequences, of which 1,762 are epitopes and 1,757 are nonepitopes. The length of sequences ranges from 6 to 30 meter. For each sequence, we extracted 13 physicochemical features. The proposed ensemble model achieved sensitivity, specificity, Gini coefficient, AUC, precision, F-score, and accuracy of 0.976, 0.959, 0.993, 0.994, 0.989, 0.985, and 97.13%, respectively. To check the consistency of the model, we carried out five-fold cross-validation and an average accuracy of 96.072% is reported. Finally, a comparative analysis of the proposed model with existing methods has been carried out using a separate validation data set, suggesting the proposed ensemble model as a better model. The proposed ensemble model will help predict novel ZIKV vaccine candidates to save lives globally and prevent future epidemic-scale outbreaks.

## 1. Introduction

ZIKV is an enveloped virus that belongs to the genus *Flavivirus* and the family Flaviviridae. It is almost similar to dengue fever and the West Nile virus because of its propagation through infected mosquito stings [1]. The World Health Organization (WHO) declared the outbreak a “public health emergency of international concern” in February 2016. To date, the shreds of evidence of ZIKV disease have been reported from 86 countries and territories [2]. The recent outbreak of ZIKV infection was reported from the Thiruvananthapuram district of the Kerala state of India in early July 2021 [3]. The majority of the people infected with ZIKV are asymptomatic. Generally, symptoms include mild fever, conjunctivitis, joint pain, muscle pain, malaise, and headache that usually last for 2–7 days. The incubation period of the virus is 3–14 days [4]. The infection shows teratogenicity, potentially causing congenital abnormalities such as microcephaly and other pregnancy-related complications such as stillbirth, preterm birth, and fetal loss [5]. In older children and adults, ZIKV infection has been reported to be the main trigger of neuropathy, Guillain–Barre syndrome, and myelitis [6].

ZIKV is a single-stranded, nonsegmented positive-sense RNA virus and has a genome of 10.7 kb, which can be translated directly into one long protein. The protein can encode three structured proteins (capsid (C), envelope (E), and membrane protein (M)) as well as seven nonstructured proteins (NS1, NS2A, NS2B, NS3, NS4A, NS4B, and NS5) [6]. The principal antigenic determinant is envelope (E) glycoprotein, which mediates the fusion and binding at virus entry. Therefore, the envelope (E) glycoprotein is a primary research target for developing antiviral therapeutics and vaccine candidates [5–7]. Although ZIKV infection is a severe and fatal disease, there is no effective vaccine and specific medicine to combat the infection. However, people need to follow certain precautions to prevent this infection, such as taking enough water to stop dehydration, use of paracetamol or analgesics, acetaminophen, and taking rest [8, 9].

Nevertheless, these measures are not enough to prevent this infectious disease. The development of a vaccine for the treatment of ZIKV is critical in the current scenario since the virus has killed a large number of people in Brazil and is spreading to other regions of the world. There is currently no preventive or therapeutic vaccination available in the market to prevent this infection [10]. Though the development of a live attenuated yellow fever vaccine (YFV) was a significant step forward, with recent developments, epitope-based vaccines are becoming more important, as the live attenuated vaccine can be deadly in immunocompromised patients [11]. Several ZIKV vaccines are presently under development to directly target the virus, with different parts of the virus serving as the basis [11]. Because infants and pregnant women are at risk of antibody-dependent enhancement (ADE) upon entry of a related *Flavivirus*, safety becomes the primary concern in developing a ZIKV vaccine [11]. The peptide vaccine is thought to be a safe platform for vaccine development. Unnecessary antigenic components can be removed by only employing the sections of a protein that can elicit an immune response. In the case of ZIKV, CD8+ T-cell activity has been proven to protect against ADE in dengue infection [12, 13]. When compared to conventional vaccines, the epitope-based vaccine has fewer side effects, is easier and less expensive to manufacture, does not contain a whole pathogen component, and takes less time to produce along with improved specificity, stability, and sustainability [13]. So to have an effective and viable vaccine against the different strains of ZIKV, it is essential to select the number of antigenic epitopes because epitope-based vaccines are considered safe [14]. Studies conducted on other Flaviviridae viruses suggest that an adaptive immune response to *Flavivirus* includes the role of neutralizing antibodies such as CD8+ and CD4+ T-cells [10, 15].

### 1.1. Motivation and Contribution

Immunoinformatics study has discovered that many conservative and highly immunogenic T-/B-cell epitopes (antigenic determinants recognized by host immune cells and capable of eliciting both humoral and cellular immunological response) on the virus antigen could be utilized as candidate vaccine targets [15]. These epitopes can induce a protective immune response against a wide range of pathogenic microorganisms.

With the advancement of machine learning techniques in biology and the growing prevalence of ZIKV infection, it is critical to establish a robust model for predicting ZIKV T-cell epitopes to design an effective and viable epitope-based peptide vaccine against this lethal virus.

Epitope-based vaccines are considered powerful alternatives to conventional vaccines due to their low production cost, less reactogenic, and allergenic responses and overcome the issues associated with using whole-organism vaccines.

This is the first study to propose a voting ensemble model based on machine learning to predict ZIKV T-cell epitopes for designing. Predictions obtained for each class (epitope or nonepitope) by the individual classifier are summed up, and the class with the majority vote is predicted. The proposed ensemble model predicts variable-length peptides, unlike CTLpred [16], where prediction of peptides up to length 9 meter is allowed. Also model shall predict epitopes directly, unlike the NetMHC [17] server, which estimates the binding capacity of a peptide sequence. The base classifiers used in the study (as discussed in Section 4.2) are trained using the physicochemical of amino acids. An odd number of classifiers have been used to avoid the occurrence of ties in the voting.

The model proposed in this study achieved 97.13% accuracy, which is promising. We carried out five-fold cross-validation to check its consistency, and it was found that its performance is almost linear with an average accuracy of 96.072%. Finally, the comparative analysis has been done with existing methods using a separate validation data set suggesting the proposed ensemble model as a better model. The proposed model will help scientists and biologists in predicting novel ZIKV vaccine candidates.

The rest of the paper is organized as follows.  Section 2 covers related work.  Section 3 details data set, feature extraction, feature selection, and target variable. The proposed ensemble model, its methodology, and machine learning classifiers used in the current study are explained in Section 4. Performance evaluation metrics are explained in Section 5. Experimental results are presented in Section 6. Discussion is done in Section 7. Conclusions drawn and directions for future work are presented in Section 8.

## 2. Related Work

The in silico approach has emerged as a promising field for epitope prediction [18]. Many in silico based studies and methods exist for the prediction of ZIKV T-cell epitopes. In their study, Alam et al. [19] obtained envelope glycoprotein and strong immunogenic T-cell epitopes of ZIKV from the protein database. They have primarily focused on MHC class 1 potential peptides. As per their study, MMLELDPPF-GLDFSDLYY and YRIMLSVHG-VLIFLSTAV are the highly dominant predicted epitopes pairs for CD8+ and CD4+ T-cells, respectively. The authors used the NETCTL_1.2 online tool [20] with a 0.95 threshold to maintain specificity and sensitivity of 0.95 and 0.90, respectively, for T-cell epitope prediction.

In their study, Dar et al. [15] retrieved 54 sequences of the ZIKV polyprotein from the NCBI website. They used a consensus sequence to predict T-cell epitope sequences that bind MHCI and MHC-II alleles utilizing the PorPred1 [21] and ProPred [22] tool, respectively. Authors later used VaxiJen 2.0 tool to calculate the antigenicity score for each epitope predicted.

Wiwanitkit and Wiwanitkit [23], in their study on Brazil-ZKV2015 ZIKV isolate (complete genome with GenBank ID: KU497555.1), have used a standard bioinformatics tool, namely SVMTriP [24]. A combination of propensity and similarity of tripeptide subsequence has been used to predict epitopes, and a sensitivity of 80.1% has been achieved.

In their study, Yadav et al. [25] predicted MHC class II promiscuous epitopes using the immunoinformatics tool ProPred [22]. The chosen MHC alleles and epitopes were molecularly modelled using the CPH model [26] and PEP-FOLD server [27, 28], respectively. Furthermore, the viral glycoprotein having YRIMLSVHG epitope bound to MHC class II allele DRB1∗01 : 01 has shown a remarkable binding score.

In their study, Kumar Pandey et al. [29] applied the combinatorial immunoinformatics technique for developing a multiepitope subunit vaccine by using structural and nonstructural proteins of ZIKV. The subunit vaccine comprises helper T lymphocyte and cytotoxic T lymphocyte epitopes with appropriate linkers and adjuvant.

In their research, Prasasty et al. [30] used immunoinformatics to find candidates for T-cell epitopes in a series of ZIKV proteomes. The authors performed mapping of candidate's T-cell epitopes using specified HLA alleles. The authors later demonstrated a clear peptide-HLA interaction for major histocompatibility complex II (MHC-II) epitopes using molecular docking.

Shahid et al. [31], in their study, have used a combination of molecular docking and immunoinformatics techniques to constitute a multiepitope-based peptide (MEBP) vaccine. The authors used the ZIKV proteome to predict T-cell (HTL and CTL) epitopes. Following prediction, authors have shortlisted strongly overlapping and antigenic epitopes with 11 HTL and 14 CTL epitopes linked to final peptides via GPGPG and AAY linkers, respectively.

On the other hand, the NetMHC server [17] based on SVM (support vector machine) and neural network classifiers predict the only binding capacity of peptides instead of a deterministic way of prediction (discrete-valued output, i.e., 1 for epitope and 0 for nonepitope). However, the CTLpred server [16] employing artificial neural network, support vector machine, and quantitative matrix techniques predict peptides in a deterministic way. Still, it can predict peptides of length up to 9 meter only.

## 3. Materials and Methods

### 3.1. Sequence Retrieval and Preparation of the Data Set

The experimentally determined ZIKV peptide sequences (epitopes and nonepitopes) were taken from IEDB [32]. The data set consists of 3,519 linear peptide sequences, of which 1,762 are T-cell epitopes and 1,757 are nonepitopes. The peptide sequences belong to both MHC I and MHC II classes. The length of sequences is in the range of 6 to 30 meters. The glimpse and structure of the data set are shown in Table 1, where column SL denotes sequence length and class column denotes the target class, that is, epitope as 1 and nonepitope as 0.

### 3.2. Feature Extraction

In the current study, we utilized the physicochemical properties of amino acids to extract features from peptide sequences. The physicochemical properties represent a feature here. We used peptides [33] and peptider [34] packages of *R* language to extract 13 features. The essential physicochemical properties, the necessary *R* packages, functions inside the package, and the notations used in the current study are listed in Table 2.

### 3.3. Feature Selection

Feature selection is a method of selecting essential features to boost model efficiency while discarding those with irrelevant information. The feature selection was performed using importance() function of the random forest algorithm available under the package FSelectorin R. The input to the algorithm is a data set of 13 features and target attributes, that is, class. The function then computes the importance of each feature using the mean decrease in accuracy and mean decrease in node impurity. In the current study, mean decrease in accuracy has been used because it is based on experiments using out-of-bag (OOB) samples and works by reducing a predictive power of feature without changing its marginal distribution. Based on the mean decrease in accuracy, 3 features are discarded out of 13 using cutoff.k function in *R*, and only the top 10 features are considered important.  Table 3 shows all the features with their importance score.  Figure 1 shows their line plot, and the following equation shows the model equation as a function of the top 10 important features to train the model:

(1) $$\begin{array}{c} \text{Class}∼f\left(F4,F6\_2,F6\_1,F8,F2,F10,F5\_1,F1,F3\right). \end{array}$$

### 3.4. Target Variable

Class is a target variable in this study with binary instances, namely epitope (1) and nonepitope (0). An epitope is a part of an antigen or foreign protein that binds to a specific antigen receptor and can stimulate an immune response. The flowchart shown in Figure 2 demonstrates how our proposed ensemble model classifies a peptide sequence as ZIKV T-cell epitope or nonepitope.

## 4. Proposed Voting Ensemble Model

Voting-based ensemble learning is an effective technique for improving the accuracy of a classifier by merging a set of base models or classifiers. All these classifiers vote for a new instance. The prediction output is a label “class” in this study based on the majority votes. We developed an ensemble-based prediction model by combining support vector machine (SVM), random forest (RF), decision tree (DT), neural network (NN), and AdaBoost classifiers (Ada). These classifiers are used as base classifiers because their performance for binary classification problems is superior to that of other classifiers.

### 4.1. Proposed Ensemble Methodology

Figure 3 depicts the methodology followed in the current study, while Figure 4 depicts the ensemble-based learning technique, which has been followed in building the ensemble model. The steps mentioned below demonstrate the methodology of our proposed ensemble model.

**Step 1 .**

Obtaining peptide sequences

The ZIKV peptide sequences (epitopes and nonepitopes) were obtained from the IEDB website in a comma separated values (CSV) format. We retrieved two CSV files, one containing epitope and other nonepitope sequences. We labelled the epitope sequences with “1's” and nonepitopes sequences with “0's” as the target class.

**Step 2 .**

Feature extraction

The two CSV files obtained in Step 1 are given as input to physicochemical property functions (as shown in Table 2) inside peptides and peptider packages of *R* that produced two separate CSV files. One file contains epitope sequences and the other contains one nonepitope sequences. Each row in the CSV file corresponds to one peptide sequence and consists of thirteen features (physicochemical property values). These two CSV files were then merged to form a final data set with a binary variable “class” as the target variable.

**Step 3 .**

Data cleaning

Data cleaning and feature selection methods are used to perform data preprocessing. We cleaned the data set before building the model to achieve precise and highly reliable information. The main focus of data cleansing in our study was to remove duplicate entries, eliminate data anomalies, and handle outliers. We found some duplicate entries of sequences and removed them as part of the data cleaning process. Outlier detection was also carried out. Any data instance that has a significant deviation from other instances is known as an outlier and can cause problems in model prediction. All the outliers were removed from the data set before carrying out feature selection and model building.

**Step 4 .**

Feature selection

Feature selection is a technique for reducing dimensionality that enhances the model performance. We used a random forest importance algorithm that selected only 10 essential features. The following formula depicts the target class and its corresponding features used in our proposed ensemble model:

(2) $$\begin{array}{c} \text{Class}∼f\left(\text{ppeptide}+\text{hydrophobicity}+\text{isoelectric point}+\cdots +\text{instability index}\right). \end{array}$$

**Step 5 .**

Classification model building using ensemble learning

In this study, we used 80% of the data set for model training to achieve better results and 20% for testing. We trained all base models (random forest, decision tree, SVM, neural network, and AdaBoost) on 80% of the total data set and combined them using the ensemble technique.

**Step 6 .**

Predictions by the voting-based ensemble method

The accuracy of the proposed ensemble model is assessed using a test data set that is 20% of the total data set. The evaluation is based on a majority vote system of five base classifiers, that is, random forest, decision tree, SVM, neural network, and AdaBoost. As a result, the proposed ensemble model combines five base classifiers and will be our final prediction model for predicting the class or type of a ZIKV peptide sequence, whether epitope or nonepitope. Since these testing tuples are predicted by voting of five base classifiers, the proposed model predicts them perfectly and gives accurate and reliable results.

### 4.2. Machine Learning Classifiers Used in the Current Study

Classifiers used for the prediction of ZIKV T-cell epitopes are listed in Table 4. Each classifier has its required package, method, and necessary tuned parameters. We performed tuning of essential parameters of all the classifiers to get a better prediction result and implemented them in *R* under the GNU-GPL (general public license). Machine learning classifiers used in the current study are described below.

#### 4.2.1. Decision Tree

The decision tree classifier predicts the target variable value (class in this study) based on the input predictor variables. It is organized in the form of a flowchart with each internal node representing a check or test on the input variable. Edges to child nodes represent an outcome of a trial, and leaf node acts as the class label. To infer decision trees, we have used rpart() function in *R*. We performed the parameter tuning of its “usesurrogate” and “maxsurrogate” parameters to improve its performance. Parameter “maxsurrogate” means the number of surrogate splits that are kept in the output. The search for surrogate splits consumes almost half of the computing time (other than setup). Parameter “usesurrogate” means how to employ surrogates in the splitting process. A value of 0 indicates that the observation is merely for display, and 1 denotes the usage of surrogates. Setting these parameters to 0, the processing time is significantly reduced since the search for surrogate splits takes up roughly half of the computing time.

#### 4.2.2. Support Vector Machine (SVM)

With the SVM classifier, we construct a hyperplane that divides the two sets (epitope or nonepitope) in the *n*-dimensional space. Here “*n*” equals the number of features of a given peptide. In *R*, the package kernlab contains the function ksvm() for the support vector machine. We improved its performance by tuning parameters “type” and “kernal” of kvsm. For better performance, we have used the radial basis kernel function (rbfdot), “Gaussian.” The “type” parameter indicates whether it is classification or regression or novelty detection. Depending on whether *y* is a factor, the default value for type is “C-svc” or “eps-svr.” It is a classification problem so we have assigned C-svc to it as “type = C-svc.” The kernel function is used in training, and prediction computes the inner product in feature space between two vector parameters.

#### 4.2.3. Random Forest

A random forest is an ensemble of decision trees. Here, the result provided by the random forest classifier is based on the majority votes of decision trees for the particular class. In *R*, the package randomForest contains a function randomForest() that returns a random forest classifier object. We performed the parameter tuning of “mtry” and “ntree” among its various parameters to improve its performance. The reason tuning of “mtry” and “ntree” has been performed in the current study that they have the biggest effect on final accuracy. The parameter “mtry” denotes the number of randomly sampled features at each division, while “ntree” represents the tree count. The random forest model used in this study achieved better performance at values 2 and 500 for “mtry” and “mtry,” respectively.

#### 4.2.4. AdaBoost

Also known as an adaptive boosting algorithm, it converts the set of weak learners to strong learners. In *R*, the package ada contains a function ada() for the AdaBoost classifier. Its performance is outstanding on discrete data, and for this reason, we tuned its type parameter “type”, which means boosting algorithm type, and assigned the value “discrete” to it to perform discrete boosting. Other values it can take are “real” for real boost and “gentle” for performing gentle boosting. For iteration parameter “iter,” we set a weight of 50 to it for efficient boosting that indicates number of boosting iterations to be performed and 0.5 to shrinkage parameter “nu” (default value of 1) for performance boosting of AdaBoost.

#### 4.2.5. Neural Network

The neural network is a robust classifier consisting of nodes, also known as neurons that are interconnected. These neurons are organized into three layers: input, hidden, and output. Every neuron is connected to every other neuron through a link, and each link is associated with a value called weight with information about an input signal. In *R*, the package nnet contains a function nnet() for the neural network classifier. The essential parameters tuned are network size as “size” and maximum iterations as “maxit.” The parameter “maxit” indicates the maximum number of iterations having a default value of 100. Parameter “size” means the total number of units in the hidden layer. Parameter “size” is set to 0 if there are skip-layer units. In this study, values of 10 and 300 have been assigned to “size” and “maxit” parameters, respectively, to achieve better results and avoid overfitting. Also, it is worth mentioning that it is recommended to set “maxit = 300” for data set consisting of 3,000 to 5,000 data instances. Setting it to a higher value can cause an overfitting problem.

## 5. Performance Evaluation Metrics

We assessed and compared the performance of the proposed ensemble model to existing models using binary classification performance metrics such as sensitivity, specificity, Gini coefficient, precision, F-score, accuracy, and AUC. These are described below.

### 5.1. Area under the Curve (AUC)

For binary classification problems, receiver operator characteristic (ROC) curve is a crucial evaluation metric. The ROC curve is a probability curve where we plot true positive rate (TPR) versus false positive rate (FPR) at different thresholds, thus effectively distinguishing signal from noise. The value of the ROC curve at the top left corner is considered as the best value compared to other values.

### 5.2. Sensitivity (Sens)

Sensitivity (Sens) is also termed as true positive rate (TPR) or recall. It is a measure of the proportion of true positive instances that the model predicted as positive. It is calculated as follows:

(3) $$\begin{array}{c} \text{sensitivity}=\frac{\text{TP}}{\text{TP}+\text{FN}}. \end{array}$$

### 5.3. Specificity (Spec)

Specificity (Spec) is also termed as true negative rate (TNR). It is a measure of the proportion of real negative instances that the model predicted as negatives. It is calculated as follows:

(4) $$\begin{array}{c} \text{specificity}=\frac{\text{TN}}{\text{TN}+\text{FP}}. \end{array}$$

### 5.4. Gini Coefficient

The Gini coefficient gives a measure of the distribution of inequality in data. The Gini coefficient ranges from 0 to 1. While value 1 denotes perfect data inequality, value 0 denotes perfect data equality. For example, given two models A and B have Gini coefficients as 0.7 and 0.5, respectively, then model A is more productive than model B and is computed as follows:

(5) $$\begin{array}{c} \text{Gini}=2*\text{ AUC}-1. \end{array}$$

### 5.5. Precision

Precision is a measure of exactness, that is, the number of correct positive instances. It is calculated as follows:

(6) $$\begin{array}{c} \text{precision}=\frac{TP}{TP+FP}. \end{array}$$

### 5.6. Accuracy

Accuracy is defined as the percentage of right predictions on test data. It is computed as follows:

(7) $$\begin{array}{c} \text{accuracy}=\frac{TP+TN}{TP+FP+TN+FN}*100. \end{array}$$

### 5.7. F-Score

It is the harmonic mean of recall and precision. It is calculated as follows:

(8) $$\begin{array}{c} F-\text{score}=\frac{2*\text{precision}*\text{recall}}{\text{precision}+\text{recall}}. \end{array}$$

## 6. Results

### 6.1. Performance Results of the Proposed Ensemble Model and Existing Classifiers

For a binary classifier, the Gini coefficient, precision, sensitivity, specificity, AUC, F-score, and accuracy are the assessment parameters defined in Section 5. We used these parameters to evaluate our proposed ensemble model's performance and compare it to existing classification models for ZIKV T-cell epitope prediction, as shown in Table 5. The model achieved AUC, sensitivity, specificity, precision, F-score, Gini coefficient, and accuracy of 0.994, 0.976, 0.959, 0.989, 0.985, 0.993, and 97.13%, respectively.  Figure 5 depicts a performance comparison chart of existing models with the proposed ensemble in terms of accuracy.  Figure 6 depicts the ROC plot of the proposed model on the testing data set with an AUC of 0.994. The obtained results demonstrate that the proposed ensemble model performs better as compared to the existing classification models when tested using the test data set.

### 6.2. *K*-Fold Cross-Validation Results of the Proposed Ensemble Model

We carried out five-fold cross-validation (CV; *k* = 5 in this study) to estimate the ability of the proposed ensemble model and assess its robustness. The data set was divided into five folds. Four folds are used to fit the model, and one fold is held out to evaluate the model.  Table 6 describes the accuracy of each run, and Figure 7 depicts the plot of accuracies recoded in five-fold CV for Zika virus T-cell epitope prediction.

The accuracy of each run as shown in Figure 7 depicts the accuracy plot as recoded in a five-fold CV for the prediction of ZIKV T-cell epitopes. The average accuracy achieved through five-fold CV is 96.072%. It is visible from the results obtained in a five-fold CV that the proposed ensemble model performs consistently on all the folds.

### 6.3. Comparison Results of the Proposed Ensemble Model with Existing Methods

A separate validation data set was used for performance validation, including eight ZIKV T-cell epitopes and five nonepitopes. These peptide sequences are neither present in the training set nor the testing set and are also called the blind data set. Suppose the performance of our proposed model on the validation data set is satisfactory; in that case, it completes the validation process, and as shown in Table 7, the results are excellent because it correctly classifies all of the peptide sequences in the validation set.

The validation results of our proposed ensemble model using validation data set were compared with the existing T-cell epitope prediction methods, that is, NetMHC and CTLpred, because these are the most frequently used methods for T-cell epitope prediction methods by scientists, biologists, and researchers. Since the NetMHC server only provides peptide-binding capacity, the proposed ensemble model is more efficient for it directly predicts whether a peptide is a ZIKV T-cell epitope or not (Table 7). CTLpred server only predicts T-cell epitopes of length up to 9 meter. As shown in Table 7, prediction by CTLpred for sequences having a length greater than 9 meter is shown as a hyphen (-), which means “unpredicted” as CTLpred cannot predict them. However, our proposed ensemble model predicts peptide sequences of any size. In addition, the CTLpred server is limited to ANN and SVM, but more powerful and efficient classifiers were used in our proposed ensemble model. The comparison results shown in Table 7 show that the proposed model performs better than existing methods.

## 7. Discussion

ZIKV disease is considered one of the devastating diseases affecting millions of lives globally, especially in the third world. In its news bulletin report [40], the WHO has reported that its global spread and recent outbreaks underline the need for research in vaccine development and its continued vigilance. Using an experimental approach to identify ZIKV T-cell epitopes is an expensive and time-consuming process. Designing vaccines based on epitopes is already showing remarkable and hopeful results. This technology plays a pivotal role in treating and preventing cancer, bacterial, viral, and other types of diseases [41, 42]. Therefore, it is high time to utilize and take advantage of rapid developments in the immunoinformatics approach. This study proposes an ensemble model for predicting ZIKV T-cell epitopes with impressive results. Its statistical performance analysis was assessed using various performance metrics such as AUC, precision, sensitivity, specificity, Gini coefficient, F-score, and accuracy. The predictive performance of positive classes (epitopes) is represented by sensitivity, while the predictive performance of negative classes is represented by specificity (nonepitopes). On the other hand, accuracy is the most crucial parameter for determining how well the proposed ensemble model predicts epitope and nonepitope classes. As a result, an excellent binary classifier has high precision, sensitivity, and accuracy. The specificity, sensitivity, and accuracy values for our proposed model are 0.976, 0.959, and 97.13%, respectively, which is promising.

## 8. Conclusion

An ensemble-based computational method was developed for predicting ZIKV T-cell epitopes in this study. Class is the target variable for epitope prediction, and the data set used in the current study is balanced with nearly equal numbers of epitopes and nonepitopes. Feature extraction of peptide sequences was performed using physicochemical properties of amino acids and feature selection with the help of a random forest importance algorithm. The proposed ensemble model was tested using performance parameters such as AUC, sensitivity, specificity, precision, F-score, Gini coefficient, and accuracy, and the values achieved were 0.994%, 0.976%, 0.959%, 0.989%, 0.985%, 0.993%, and 97.13%, respectively. Through rigorous experiments, it was discovered that the proposed ensemble model outperforms the existing models used in this study, such as random forest, decision tree, SVM, neural network, and AdaBoost.

Furthermore, the performance of the proposed ensemble model is almost linear as measured by five-fold cross-validation with an average accuracy of 96.072% recorded. Finally, the validity of the proposed ensemble model was tested using a validation data set containing new peptide sequences. These new peptide sequences are neither present in training nor in the testing data set, where 100% accuracy was achieved. The proposed ensemble model will help biologists and scientists predict novel ZIKV vaccine candidates in less time and in a cost-effective manner so as to save lives globally and prevent future epidemic-scale outbreaks. Predicting novel ZIKV vaccine candidates through wet lab experiments is an expensive task and takes a lot of time. Nevertheless, it is pertinent to mention that some spaces can be improved, like exploring more properties of amino acids and using other machine learning classifiers. Therefore, our future work will focus on enhancing the robustness and accuracy of prediction by exploring more machine learning classifiers and the physicochemical properties of amino acids.

## Figures and Tables

**Figure 1:** Feature importance line plot.

**Figure 2:** Workflow for classification of peptide sequences.

**Figure 3:** Methodology used.

**Figure 4:** The proposed ensemble model for ZIKV T-cell epitope prediction.

**Figure 5:** Comparison chart of existing models with the proposed model.

**Figure 6:** ROC plot of the proposed ensemble model.

**Figure 7:** Five-fold cross-validation results of the proposed ensemble model.

**Table 1:** Snapshot of the data set.

Peptide sequence	SL	F1	F2	F10	F11	Class
GSLQLLAIE	9	184.4444	−0.74222	−0.56222	3	0
EEQRYTCHVQHEGLPKPLTLRW	22	66.36364	2.643182	−0.08955	4	0
LQSNGWDRLKRMAVS	15	78	2.785333	−0.07	4	1
YKYKVVKIEPLGVA	14	125	−0.06929	−0.12429	2	0
GDTLKECPLKHRAWNSFL	18	70.55556	1.928889	−0.02667	5	1
HMCDATMSY	9	11.11111	1.3	−0.18	4	1
KAFEATVRGAKRMAV	15	65.33333	1.915333	−0.62	6	1
CKRGIKSGS	9	43.33333	2.748889	0.385556	5	0
WASRELERF	9	54.44444	3.868889	−0.46222	2	0
AVRHFPRIW	9	86.66667	2.046667	−0.09444	1	0

**Table 2:** Physicochemical properties used in the current study.

Sr. no.	Property name	Package	Function name	Notation
1	Aliphatic index	Peptides	aIndex (seq)	F1
2	Potential protein interaction index	Peptides	Boman (seq)	F2
3	Instability index of a protein sequence	Peptides	instaIndex (seq)	F3
4	Probability of detection of a peptide	Peptider	Ppeptide (x, libscheme, N)	F4
5	Hydrophobic moment (1) Protein rotational angle a-helix = 100 (2) Protein rotational angle b-sheet = 160	Peptides	hmoment (seq, angle)	F5_1, F5_2
6	Molecular weight (1) Monoisotopic = false (2) Monoisotopic = true	Peptides	Mw (seq, monoisotopic)	F6_1, F6_2
7	Theoretical net charge at 9 pKa scales	Peptides	charge	F7
8	Hydrophobicity index	Peptides	Hydrophobicity	F8
9	Isoelectric point	Peptides	pI	F9
10	Kidera factors	Peptides	kideraFactors	F10
11	Amino acid composition	Peptides	aaComp	F11

**Table 3:** Feature importance score.

Feature	Score
F4	60.53
F6_2	52.03
F6_1	51.95
F8	46.15
F2	44.18
F10	43.43
F9	42.25
F5_1	41.69
F1	40.87
F3	39.49
F5_2	38.08
F7	36.36
F11	30.52

**Table 4:** Machine-learning classifiers were used in the current study.

Sr. no.	Classifier	*R* package	Tuned parameters
01	Decision trees [35]	rpart	maxsurrogate = 0, usesurrogate = 0
02	Neural network [36]	nnet	Size = 10, maxit = 100
03	Support vector machine [37]	ksvm	kernel = “rbfdot,” type = C-svc”
04	AdaBoost [38]	ada	Iter = 50, type = “discrete,” nu = 0.5
05	Random forest [39]	randomForest	ntree = 500, mtry = 2

**Table 5:** Performance comparison of existing models with the proposed ensemble.

Model	Gini	Precision	F-score	AUC	Sensitivity	Specificity	Accuracy (%)
Random forest	0.905	0.963	0.958	0.952	0.953	0.921	94.29
Neural network	0.990	0.936	0.951	0.973	0.948	0.963	96.52
AdaBoost	0.988	0.985	0.963	0.994	0.942	0.972	95.24
Decision tree	0.987	0.972	0.972	0.993	0.972	0.938	96.19
SVM	0.912	0.979	0.975	0.995	0.972	0.956	96.67
Proposed ensemble model	0.993	0.989	0.985	0.994	0.976	0.959	97.13

**Table 6:** Five-fold cross-validation.

Fold	Accuracy
1	96.27
2	95.28
3	97.52
4	96.49
5	94.80

**Table 7:** Validation results of the proposed ensemble model and its comparison with existing methods.

Peptide sequence	Actual target	Comparison with NetMHC		Comparison with CTLpred	
		Binding capacity by NetMHC	Predictions by the proposed model	Predictions by CTLpred	Predictions by the proposed model
NSFVVDGDT	Epitope	49	1	Epitope	1
VREDYSLECDPAVIG	Epitope	25	1	—	1
AQMAVDMQT	Epitope	3.9	1	Epitope	1
FVVDGDTLKECPLKH	Epitope	2.2	1	—	1
GEAYLDKQ	Epitope	75	1	Nonepitope	1
GPSLRSTTASGRVIE	Epitope	34	1	—	1
MEIRPRKEPESNLVR	Epitope	65	1	—	1
TRGPSLRST	Epitope	7.2	1	Epitope	1
MLRIINARG	Non epitope	3.4	0	Nonepitope	0
IQIMDLGHMATC	Non epitope	56	0	—	0
LVTCAKMQ	Non epitope	80	0	Nonepitope	0
LGGFGSL	Non epitope	78	0	Epitope	0
VVVLGSQERIN	Non epitope	34	0	—	0

## Data Availability

Data are available on request to the corresponding author.
